# miR-539 Targeting SNAI2 Regulates MMP9 Signaling Pathway and Affects Blood-Brain Barrier Permeability in Cerebrovascular Occlusive Diseases: A Study Based on Head and Neck Ultrasound and CTA

**DOI:** 10.1155/2021/5699025

**Published:** 2021-11-27

**Authors:** Hui Li, Guochao Han, Dongruo He, Ying Wang, Yuan Lin, Tianyu Zhang, Jiandong Wang, Youli Du, Gang Li, Yuguang Wang, Jiexin Zhou, Bo Liu

**Affiliations:** ^1^Neuroelectrophysiology Department, The Second Affiliated Hospital of Qiqihar Medical College, Qiqihar 161000, China; ^2^Department of Ultrasound, The Second Affiliated Hospital of Qiqihar Medical College, Qiqihar 161000, China; ^3^CT Department, The Second Affiliated Hospital of Qiqihar Medical College, Qiqihar 161000, China; ^4^Department of Neurology, The Second Affiliated Hospital of Qiqihar Medical College, Qiqihar 161000, China; ^5^Department of Interventional Therapy, The Second Affiliated Hospital of Qiqihar Medical College, Qiqihar 161000, China; ^6^Department of Fundamentals, Qiqihar Medical College, Qiqihar 161000, China

## Abstract

This study aimed to explore the expression level of miR-539 in the blood-brain barrier permeability induced by cerebrovascular occlusion and its mediated mechanism. Altogether, 48 patients with cerebral vascular occlusion lesions from March 2018 to June 2020 were collected. The expression level of miR-539 in the peripheral blood serum of the subjects was analyzed by qRT-PCR, and the participants were divided into two groups according to the results of head and neck ultrasound and CTA hemodynamics. The MCAO model of cerebral ischemia was established in rats, and the expression level of miR-539 was detected by qRT-PCR in brain tissues of different groups of rats. The effects of miR-539 on the permeability of blood-brain barrier were investigated by intraventricular injection of agomiR-539 and antagomir-539. The model of blood-brain barrier was established by culturing brain microvascular endothelial cells and pericytes in vitro, and the changes of miR-539 expression level and permeability after glucose and oxygen deprivation were detected. The expression level of SNAI2/MMP9 signaling pathway protein in cells was detected by Western blot. Compared with the healthy control group, the expression level of miR-539 in peripheral blood of patients with cerebrovascular occlusive disease decreased significantly, and the expression level of miR-539 in the MCAO rat model decreased and affected the permeability of blood-brain barrier. Glucose and oxygen deprivation treatment in brain microvascular endothelial cells can lead to downregulation of miR-539 expression and affect cell permeability. miR-539 in brain microvascular endothelial cells can target and bind to SNAI2 and participate in the regulation of endothelial cell permeability by affecting the SNAI2/MMP9 signaling pathway. The results of this study suggested that circulating miR-539 in peripheral blood may be a potential marker for predicting blood-brain barrier permeability after ischemic stroke. More detailed studies are needed to determine its diagnostic value.

## 1. Introduction

At present, it has been reported that ischemic stroke accounts for 60%–80% of stroke cases in China [1]. Acute ischemic stroke patients with arterial occlusion have a poor response to intravenous injection of recombinant tissue plasminogen activator, bringing a high possibility of deterioration and poor prognosis after 24 h [2]. Blood-brain barrier refers to the barrier structure between plasma and brain cells formed by brain capillary endothelial cells, astrocytes, and pericytes. It prevents almost all macromolecules and 95% of small molecules from entering the brain, limiting the entry of pathogens and toxic substances, maintaining the steady state of brain microenvironment and ensuring the normal function of the nervous system [3, 4]. However, cerebral vascular occlusive disease leads to acute ischemic stroke, which leads to the destruction of blood-brain barrier and the increase of permeability of blood-brain barrier by mediating energy failure. The excitotoxicity, inflammatory immune response, oxidative stress, and apoptosis would be increased, leading to a series of complications [5, 6]. According to reports, acute cerebral ischemic stroke is caused by mediation. It has been found that the abnormal expression of NADPH oxidase [7] and inflammatory pathway-related transcription factor NF-*κ*B [8] plays an important role in cerebral ischemia-reperfusion injury. But the detailed mechanism has not been reported.

Previous studies have found that overexpression of miRNA-125a-5p in brain endothelial cells can lead to thicker and more continuous junction complex formed by VE-cadherin and ZO-1, thus increasing the barrier function of cerebrovascular endothelial cells [9]. At present, it has been found that many miRNAs are significantly differently expressed in ischemic lesions, which can mediate different biological functions. It is found that there are different miRNA expressions in different blood-brain barrier cells, and some studies show that some miRNAs can participate in controlling endothelial cell function and blood-brain barrier permeability. Reijerkerk and others found that a large number of miRNAs were downregulated in the microvascular endothelium of the brain with impaired blood-brain barrier function, while the enhancement of blood-brain barrier function was usually accompanied by an increase of a series of miRNAs, including miR-125a-5p, miR-126-3p, and miRNA-155 [9–11]. At present, it has been found that miR-539 plays an important role in many tumors, including glioma, liver cancer, and colorectal cancer [12, 13]. In addition, it was found that the expression of miR-539 could also be significantly decreased in the mouse model of cerebral ischemia/reperfusion injury [14], but the related mechanism of the change of miR-539 permeability in blood-brain barrier is still unclear. At present, a large number of studies have reported that head and neck ultrasound and CTA could significantly improve the diagnostic rate of ischemic stroke and can also be used to judge whether the permeability of blood-brain barrier is damaged according to the obtained hemodynamic data. Therefore, this study aimed to explore the mechanism of miR-539 affecting blood-brain barrier permeability in cerebrovascular occlusive diseases by combining the cerebral hemodynamic indexes obtained by head and neck ultrasound and CTA.

## 2. Materials and Methods

### 2.1. Research Participants

From March 2018 to June 2020, a total of 48 patients were obtained, including 31 males and 17 females. They were aged 35–52 years, with an average age of 40.5 ± 7.2 years. All patients were diagnosed with cerebral vascular occlusive disease by carotid ultrasound, carotid magnetic resonance angiography, computed tomography angiography (CTA), and/or digital subtraction angiography (DSA). The informed consent forms were obtained from all patients or their families. Exclusion criteria: (1) patients with a history of surgery and brain trauma, (2) patients with vascular malformation, (3) patients with Takayasu arteritis and intracranial infection, (4) patients with acute and chronic infections, and (5) patients with the history of myocardial infarction and thromboembolism. The control group consisted of 48 healthy people with normal physical examination results. This research has been approved by the hospital ethics committee. All patients were informed of the experimental purpose and research plan before collecting blood and signed the informed consent form.

### 2.2. Detection of miR-539 in Peripheral Blood

A total of 2 ml of peripheral venous blood (EDTA) was collected from all the subjects and then stored in a refrigerator at 4°C. Samples were sent to the laboratory for qPCR detection within 4 h. Total RNA was extracted by TRIzol (Invitrogen); then, cDNA was synthesized by miRNA qRT-PCR SYBR (Clontech) kit, amplified according to the primer sequence given in Table 1, and then quantitatively detected in a fluorescence quantitative PCR instrument (Bio-Rad). The reaction conditions are 95°C for 15 min, 95°C for 5 s, 55°C for 5 s, and 70°C for 30 s. The relative expression of miR-539 was calculated by 2^−*δδCT*^ with U6 as internal reference.

### 2.3. Head and Neck Ultrasound and CTA Examination

Head and neck ultrasound and CTA were used to diagnose cerebral vascular occlusive disease in patients, and whether the permeability of blood-brain barrier enhanced was judged according to different hemodynamic parameters such as cerebral blood flow (CBF), cerebral blood volume (CBV), mean transit time (MTr), and permeability surface (PS).

### 2.4. Establishment of the MCAO Model of Cerebral Ischemia

Altogether, 24 adult SD rats (250 g) were randomly divided into the operation group and sham operation group, with 12 rats in each group. Rats were injected with 1% pentobarbital sodium intraperitoneally at a dose of 40 mg/kg. They were fixed on the operating table in supine position. After routine disinfection and skin preparation, the midline incision was made, and the muscles and fascia were separated along the inner edge of sternocleidomastoid muscle. The left common carotid artery, external carotid artery, and internal carotid artery were separated and clamped, respectively. The trunk of external carotid artery was separated, its branches were blocked with electrocoagulation pen, and cutoff after the distal end was ligated. A V-shaped small opening was made in the stump of the external carotid artery with ophthalmic scissors. The pretreated thread plug was carefully inserted from the incision to the direction of the common carotid artery and carefully inserted 17-18 mm to the beginning of the middle cerebral artery. After operation, the cerebral cortex blood flow was monitored by a laser speckle blood flow imager. If the cerebral cortex blood flow decreased by 70%–80%, the model could be used by rats.

### 2.5. Injection of agomiR-539 and antagomiR-539 into Lateral Ventricle

agomiR-539 and antagomiR-539 used in the experiment were purchased from Sangon Biotech (Shanghai) Co., Ltd. The method of lateral ventricle injection referred to the experimental method in previous published articles [15]. The rats were fixed in the prone position after full anesthesia. agomiR-539 and its negative control and antagomiR-539 and its negative control were dissolved in 5 *μ*l PBS at 0.5 nmol/*μ*l and 1 nmol/*μ*l, respectively. Then, they were injected into the right lateral ventricle of rats according to different injection sites (1 mm at the tail; 2.5 mm outside the midline; 3.5 mm deep on the skull surface).

### 2.6. Evans Blue Leakage Test

The experiment referred to the experimental method in the previously published article [16]. Before the experiment, 2% Evans blue solution (Sigma-Aldrich) was prepared with normal saline, which was injected into MCAO rats by tail vein at a dose of 4 ml/kg 18 h after the model was successfully established. Six hours after injection, rats were fully anesthetized and perfused with PBS to remove Evans blue dye remaining in blood vessels. The rat cerebral hemispheres were homogenized in 50% trichloroacetic acid solution and centrifuged at 20000 g, at 4°C for 20 min. After centrifugation, the supernatant was collected and mixed with absolute ethyl alcohol in a ratio of 1 : 3. Evans blue extravasation was quantified by measuring fluorescence intensity at 620 nm.

### 2.7. Cell Line Culture

The rat brain microvascular endothelial cell line (RBMVEC) was purchased from Otwobio Biotech Inc. (Guangzhou) (HT-X2348), and the rat microvascular pericytes were purchased from Procell Life Science and Technology Co., Ltd. (CP-R187) and cultured according to the instructions. The endothelial cell culture medium (ScienCell) and pericyte complete culture medium (Procell) were used for cell culture until the cell density increased to 80%–90%.

### 2.8. FITC-Dextran Permeability Test

Previous studies have reported that the permeability of the blood-brain barrier model in vitro can be evaluated by measuring the permeability of FITC-dextran (Sigma-Aldrich) with molecular weight of 40,000 [15]. The specific experimental method FITC- dextran assay buffer containing 100 *μ*g/mL was added into the upper chamber of the model, cultured for 0, 30, 60, and 120 min, and then 50 *μ*l of culture was taken out from the lower chamber.

### 2.9. agomiR-539 and antagomiR-539 Transfected Cells

RBMVEC cells were inoculated in a 24-well plate and transfected when the density increased to 70–80%. According to the instructions, 100 nM agomiR-539, antagomiR-539, or their corresponding 200 nM negative control were added to regulate the expression level of miR-539 in the cells using Lipo 2000.

### 2.10. Detection of Double Luciferase Reporter Gene

The downstream target molecules that miR-539 in web analytics may bind to were analyzed by TargetScan bioinformatics. The results showed that miR-539 may have a binding site with SNAI2. Therefore, 293T cells and a double luciferase reporter gene detection kit were used in the experiment. By constructing miR-539 mimics, miR-539 NC, and double luciferase pmirGLO vector (Guangzhou Saicheng Biotechnology Co., Ltd.), the relative light unit values of different samples were measured by the BioSpectrum chemiluminescence analyzer, and the relative activation degree of SNAI2 was calculated.

### 2.11. Western Blot

RIPA lysate (Solarbio) and protease inhibitor PMSF (Solarbio) with a final concentration of 1 mM were added into the cells, and then, the total protein of the cells was extracted by centrifugation. The total protein concentration was tested by the BCA method, the final loading protein concentration was adjusted to 5–10 *μ*g/*μ*l, the sample was loaded, and 10% SDS-PAGE separation gel was applied for gel electrophoresis. The target protein was transferred to PVDF membrane by the semiwet transfer method, sealed with 5% skimmed milk powder for 1 h, and then added with SIRT1 (60303-1-Ig, Proteintech, 1 : 4000) and MMP9 (10375-2-AP, Proteintech, 1 : 1000) primary antibody diluent at 4°C overnight. After being washed with 0.1% PBST buffer for 3 times, the corresponding HRP-labeled secondary antibody (SA00001-1/2, Proteintech, 1 : 5000) was added and incubated at room temperature for 1 h and then washed with 0.1% PBST buffer for 3 times. ECL chemiluminescence solution (Solarbio) was evenly dripped on PVDF membrane, and the expression of protein was analyzed by ImageJ.

### 2.12. Statistical Analysis

All data in this study were statistically analyzed by SPSS 24.0. The experimental results of counting data were expressed by mean ± standard deviation (*x*  ± *s*). The *t*-test was used for the comparison between the two groups, and one-way ANOVA was used for the comparison among different treatment groups. The difference was statistically significant when *P* < 0.05.

## 3. Results

### 3.1. miR-539 in Peripheral Blood of Patients with Cerebrovascular Occlusive Disease Decreased Significantly

miR-539 in peripheral blood plasma of two groups was detected by qRT-PCR. The results showed that the expression level of miR-539 in peripheral blood of patients with cerebrovascular occlusive disease was significantly lower than that of normal people (Figure 1(a)). Furthermore, the blood-brain barrier permeability of patients with cerebrovascular occlusive disease was detected by head and neck ultrasound and CTA (Figures 1(b)–1(c)). According to the results, the patients were grouped into increased permeability and unchanged permeability. It was also found that the expression level of miR-539 in peripheral blood of patients with increased blood-brain barrier permeability was also lower than that of patients with unchanged permeability (Figure 1(d)).

### 3.2. miR-539 Decreased in the MCAO Rat Model and Affected the Permeability of Blood-Brain Barrier

qRT-PCR experiment was carried out by constructing the MCAO rat model of cerebral ischemia and taking brain tissues of different groups of rats around infarction. The result was consistent with the results in patients' peripheral blood. The expression level of miR-539 in brain tissues around infarction in rats was significantly lower than that in the sham operation group (Figure 2(a)). The Evans blue leakage test showed that the permeability of blood-brain barrier increased significantly after acute occlusive hypoxia in rat brain tissue (Figure 2(b)), while agomiR-539, antagomiR-539, and their corresponding negative controls were injected into lateral ventricle, which showed that agomiR-539 could significantly reverse the increase of barrier permeability caused by acute occlusive disease (Figure 2(c)).

### 3.3. miR-539 in Brain Microvascular Endothelial Cells Can Bind to SNAI2 in a Targeted Manner

TargetScan biological information was used to analyze the downstream target molecules that miR-539 in web analytics might bind to, and the analysis results showed that miR-539 might have an interaction site with SNAI2 (Figure 3(a)), which was also verified by luciferase experiment results (Figure 3(b)). On this basis, agomiR-539 was transfected into brain microvascular endothelial cells, and Western blot results showed that overexpression of miR-539 could significantly inhibit the expression level of SNAI2 protein (Figure 3(c)).

### 3.4. miR-539 Participated in the Regulation of Endothelial Cell Permeability by Affecting SNAI2/MMP9 Signaling Pathway

Previous studies showed that SNAI2 can affect cell permeability by affecting matrix metalloproteinase expression. The specific mechanism on how miR-539 affects cell permeability was further explored in this experiment. It was found that miR-539 overexpression can significantly reduce cell permeability, while SNAI overexpression can reverse this effect (Figure 4(a)). The effect of miR-539 overexpression on matrix metalloproteinase was detected by Western blot experiment. The results showed that miR-539 overexpression significantly inhibited MMP9 expression (Figure 4(b)), which is also depended on SNAI2 expression, suggesting that miR-539' s effect on MMP9 expression level and endothelial cell permeability was mediated by SNAI2.

## 4. Discussion

Blood-brain barrier is mainly composed of brain microvascular endothelial cells in the nonperforated layer, which plays an important role in regulating the permeability of blood-brain barrier by forming a complex and compact structure with peribrain cells [17, 18]. An increasing number of studies have shown that the damage of the integrity and function of blood-brain barrier can lead to corresponding brain diseases. The decrease of blood-brain barrier function has been confirmed as an early event of multiple sclerosis and amyotrophic lateral sclerosis [19]. Among them, the changes of blood-brain barrier permeability have been widely studied in acute cerebral ischemia/reperfusion. It is found that ischemia/reperfusion significantly increases the permeability of blood-brain barrier and further aggravates brain injury caused by vascular brain edema [20]. In this study, by analyzing the expression level of miR-539 in peripheral blood of patients with cerebrovascular occlusive disease and healthy control group, it was found that the expression level of miR-539 decreased significantly in patients with cerebrovascular occlusive disease. On this basis, the results of head and neck ultrasound and CTA showed that about 43.7% of patients with cerebrovascular occlusive disease were accompanied by increased blood-brain barrier permeability, and the expression of miR-539 in peripheral blood of patients with increased blood-brain barrier permeability was lower than that of the unchanged patients, suggesting that miR-539 may play an important role in the change of blood-brain barrier permeability caused by cerebrovascular occlusive disease. In this study, the MCAO rat model with cerebral ischemia was constructed, and the brain tissues in the infarct periphery of different groups of rats were taken. It was found that the expression level of miR-539 in the brain tissues of ischemic rats also decreased, accompanied by a significant increase in Evans blue leakage, which further explained the influence of miR-539 on the permeability of blood-brain barrier.

In addition, Lopez-Ramirez and others [10] also proved that miRNA-155 participates in the regulation of cerebrovascular endothelial barrier function by targeting cell-cell complex molecules. All the above results suggested that miRNA participated in the regulation of cerebrovascular endothelial barrier by regulating the structural and functional integrity of endothelial cells. On this basis, the downstream target genes that miR-539 may bind to were detected, and we found that miR-539 may bind to SNAI and participate in the regulation of matrix metalloproteases (MMPs) in endothelial cells. Under normal circumstances, vascular endothelial cells with complete cell structure and function can secrete vascular endothelial growth factor (VEGF) and synthesize MMPs, which can promote the proliferation and invasion of vascular endothelial cells, mediate the formation of neovascular lumen, and have a certain protective effect on cerebrovascular cells and nerve cells. However, in recent years, it has been found that the hematoma formed after cerebral hemorrhage can quickly stimulate the production of a large number of MMP9, accelerate the production of edema, and intensify the destruction of nerve cells and brain cells [21]. In this study, it was found that miR-539 with high expression inhibited the activation of the MMP9-related signaling pathway and restored the permeability of vascular endothelial cells by binding to SNAI2 and reducing its expression.

## 5. Conclusion

In conclusion, the expression level of circulating miR-539 in peripheral blood of patients with cerebrovascular occlusive disease was significantly decreased, accompanied by a significant increase in permeability of blood-brain barrier, and the overexpression of miR-539 in the MCAO model of rats could reverse the effect caused by acute ischemia and hypoxia. In vitro cell experiments confirmed that miR-539 affected the expression level of MMP9 by targeting SNAI2, thus participating in the permeability regulation of blood-brain barrier composed of brain microvascular endothelial cells.

However, there are still some limitations in this study, and the results of this study have not been applied to the MCAO mouse model to explore the influence of miR-539 overexpression on blood-brain barrier in vivo. Moreover, although the results of this study suggested that circulating miR-539 in peripheral blood may be a potential marker for predicting blood-brain barrier permeability after ischemic stroke, more and more detailed studies are needed to determine its diagnostic value [22, 23, 24].

## Figures and Tables

**Figure 1:** The expression level of miR-539 in peripheral blood of patients with cerebrovascular occlusive disease decreased significantly. (a) Comparison of miR-539 expression level in peripheral blood between the healthy control group (*n* = 48) and patients with cerebrovascular occlusive disease (*n* = 48). (b) CTA examination results of patients with left common carotid artery (left) and right common carotid artery (right) occlusion. (c) Ultrasound hemodynamics of head and neck in patients with left common carotid artery (left) and right common carotid artery (right) occlusion. (d) miR-539 expression level in peripheral blood of patients with unchanged blood-brain barrier permeability (*n* = 27) and elevated blood-brain barrier permeability (*n* = 21).

**Figure 2:** The expression level of miR-539 in the MCAO rat model decreased and affected the permeability of blood-brain barrier. (a) miR-539 expression level in brain tissue around infarction in the sham operation group and MCAO rats. (b) Evans blue leakage level in midbrain tissue of the sham operation group and MCAO rats. (c) Evans blue leakage level in midbrain tissue of rats after lateral ventricle injection of agomiR-539, antagomiR-539, and their corresponding negative control in the MCAO mouse model.

**Figure 3:** Targeted binding of miR-539 to SNAI2 in brain microvascular endothelial cells. (a) Analysis of the binding target of miR-539 and SNAI2 by TargetScan biological information. (b) Luciferase experiment results verifying that miR-539 bound to SNAI2. (c) Detection of the influence of miR-539 overexpression on SNAI2 protein expression level by Western blot.

**Figure 4:** miR-539 participating in regulating endothelial cell permeability by affecting the SNAI2/MMP9 signaling pathway. (a) The permeability of miR-539 overexpression and SNAI2 overexpression to vascular endothelial cells during the culture of brain microvascular endothelial cells. (b) Western blot test used to detect the effects of miR-539 overexpression and SNAI overexpression on SNAI and MMP9 expression level.

**Table 1:** Primer sequence of fluorescence quantitative PCR amplification.

Amplified gene		Primer sequence
miR-539	Forward	5′-CGGCGGGGAGAAATTATCCT-3′
	Reverse	5′-GTGCAGGGTCCGAGGT-3′

U6	Forward	5′-GCGCGTCGTGAAGCGTTC-3′
	Reverse	5′-GTGCAGGGTCCGAGGT-3′

## Data Availability

The datasets used and/or analyzed during the current study are available from the corresponding author upon request.
